# Screening and Analysis of Key Genes in miRNA-mRNA Regulatory Network of Membranous Nephropathy

**DOI:** 10.1155/2021/5331948

**Published:** 2021-11-16

**Authors:** Yawei Hou, Yameng Li, Yichuan Wang, Wenpu Li, Zhenwei Xiao

**Affiliations:** ^1^School of Traditional Chinese Medicine, Shandong University of Traditional Chinese Medicine, Jinan, China; ^2^Affiliated Hospital of Shandong University of Traditional Chinese Medicine Nephrology, Jinan, China; ^3^Shandong University of Traditional Chinese Medicine, Jinan, China

## Abstract

**Background:**

MicroRNAs (miRNAs) are confirmed to participate in occurrence, development, and prevention of membranous nephropathy (MN), but their mechanism of action is unclear.

**Objective:**

With the GEO database and the use of bioinformatics, miRNA-mRNA regulatory network genes relevant to MN were explored and their potential mechanism of action was explained.

**Methods:**

The MN-related miRNA chip data set (GSE51674) and mRNA chip data set (GSE108109) were downloaded from the GEO database. Differential analysis was performed using the GEO2R online tool. TargetScan, miRTarBase, and StarBase databases were used to predict potential downstream target genes regulated by differentially expressed miRNAs, and the intersection with differential genes were taken to obtain candidate target genes. According to the regulatory relationship between miRNA and mRNA, the miRNA-mRNA relationship pair was clarified and Cytoscape was used to construct a miRNA-mRNA regulatory network. WebGestalt was used to conduct enrichment analysis of the biological process of differential mRNAs in the regulatory network; FunRich analyzes the differential mRNA pathways in the miRNA-mRNA regulatory network. And the STRING database was used to construct a PPI network for candidate target genes, and Cytoscape visually analyzes the PPI network.

**Results:**

Experiments were conducted to screen differentially expressed miRNAs and mRNAs. There were 30 differentially expressed miRNAs, including 22 upregulated and 8 downregulated; and 1267 differentially expressed mRNAs, including 536 upregulated and 731 downregulated. Using TargetScan, miRTarBase, and StarBase databases to predict the downstream targets of differentially expressed miRNAs, 2957 downstream target genes coexisting in the 3 databases were predicted to intersect with differentially expressed mRNAs to obtain 175 candidate target genes. Finally, 36 miRNA-mRNA relationship pairs comprising 10 differentially expressed miRNAs and 27 differentially expressed mRNAs were screened out, and the regulatory network was constructed. Further analysis revealed that the miRNA regulatory network genes may be involved in the development of membranous nephropathy by mTOR, PDGFR-*β*, LKB1, and VEGF/VEGFR signaling pathways.

**Conclusion:**

The miRNA regulatory network genes may participate in the regulation of podocyte autophagy, lipid metabolism, and renal fibrosis through mTOR, PDGFR-*β*, LKB1, and VEGF/VEGFR signaling pathways, thereby affecting the occurrence and development of membranous nephropathy.

## 1. Introduction 

Membranous nephropathy (MN) is a common pathological type of adult nephrotic syndrome. Its pathological manifestations are characterized by the formation of immune complexes under the epithelial cells of the outer visceral layer of the glomerular basement membrane and diffuse thickening of the glomerular basement membrane. The clinical manifestations are massive proteinuria, hypoalbuminemia, edema, and dyslipidemia. MN accounts for about 20% to 37% of adult nephrotic syndrome, and about 1/3 of patients eventually develop end-stage renal disease [1]. 75%–80% of MN are idiopathic membranous nephropathy (IMN), and 20%–25% are secondary membranous nephropathy or atypical membranous nephropathy. The main causes of the latter are systemic lupus erythematosus, hepatitis B virus, use of NSAIDs, and malignant tumors [2]. Studies have shown a 13% increase in the risk of membranous nephropathy in China every year, which may be related to environmental pollution [3]. A single-center study in Beijing showed that, from 2003 to 2012, the incidence of IMN in primary glomerular disease increased from 16.8% to 29.35%, and the proportion of young patients suffering from early primary membranous nephropathy increased significantly [4]. In the United States, the incidence of MN is estimated to be about 12 per million per year, with an average age between 50 and 60 years old, and the ratio of males to females is 2 : 1 [5–7]. In the United States, the incidence of ESRD caused by MN is about 1.9 per million per year [5]. In clinical observations, it was found that about 1/3 of patients with primary membranous nephropathy will be completely relieved naturally, while another 1/3 of patients will develop lifelong proteinuria while retaining kidney function for a long time, leaving 1/3 of patients will progress to end-stage renal disease [8]. Membranous nephropathy seriously endangers human health and brings a heavy economic burden to individuals and society. Therefore, early detection of the disease, early diagnosis, and appropriate treatment play a vital role in preventing or delaying the deterioration of membranous nephropathy.

Renal biopsy is the gold standard for the diagnosis of membranous nephropathy. However, because it is a traumatic operation and has certain technical requirements for physicians, and renal biopsy cannot be performed in some patients due to various reasons, there are certain limitations in clinical applications. Therefore, exploring the potential regulatory mechanism of MN and identifying new potential biomarkers and drug target genes have important guiding significance for subsequent clinical diagnosis and treatment.

MicroRNA is a type of endogenous noncoding small-molecule single-stranded RNA widely found in eukaryotes. It usually consists of 21–25 nucleotides and is highly conserved. It does not have an open reading frame itself. It participates in post-transcriptional gene regulation, affects the pathophysiological process of the body, and is related to cell development, differentiation, proliferation, apoptosis, immune regulation, tumorigenesis, etc. [9]. The study [10] found that, compared with the healthy group, the expression of miRNA-186 in the kidney tissue of patients with membranous nephropathy was significantly downregulated, and in vitro experiments proved that miRNA-186 via Toll-like receptor 4 (TLR4), P2X7, and caspase-3 participates in podocyte apoptosis, leading to increased basement membrane permeability, which in turn leads to membranous nephropathy. The study [9] found that, compared with healthy persons, increased levels of miRNA-193a were found in the urine of membranous nephropathy patients and are associated with an increase in urinary protein levels, thus increasing the severity of the disease. In addition, overexpression of miRNA-193a often indicates poor prognosis. However, there are few reports about the miRNA-miRNA regulatory network and the deep molecular mechanism of MN, especially the miRNA-mediated regulatory mechanism and the molecular network involved in the prevention and treatment of MN are still unclear. Hence, the experiment intends to use the MN-related miRNA and mRNA expression data sets in the GEO database to construct a miRNA-mRNA regulatory network using bioinformatics methods, screen key miRNA-mRNA regulatory relationship pairs, and analyze target functions and related signal pathways to explore their mechanism of action and provide important theoretical references and scientific basis for early diagnosis and targeted therapy of MN.

## 2. Materials and Methods

### 2.1. Design

Molecular bioinformatics research.

### 2.2. Time and Place

From July 2021 to August 2021, in the nephrologist's office of the Eastern District of Shandong University of Traditional Chinese Medicine Affiliated Hospital.

### 2.3. Data Source

The microarray data of miRNA expression profile and mRNA expression profile related to MN were retrieved from the GEO (Gene Expression Omnibus) database of NCBI (Table 1). Screening criteria: kidney samples from MN patients and healthy people are included, and cell lines or animal models are excluded. Finally, the miRNA expression data set GSE5167 and the mRNA expression data set GSE108109 that meet the requirements were downloaded. The data set GSE51674 was based on the platform GPL10656 and contained 16 kidney tissue samples, including 6 patients with membranous nephropathy, with an average age of 63.8 years, and 6 male patients; and there were 4 healthy patients with an average age of 38 years, 3 males and 1 female. The data set GSE108109 was based on the platform GPL19983 and contained 111 kidney tissue samples, including 6 healthy people and 44 membranous nephropathy patients.

### 2.4. Methods

#### 2.4.1. Data Processing and Differential Expression Analysis

The online analysis tool GEO2R (https://www.ncbi.nlm.nih.gov/geo/geo2r/) from NCBI's GEO online analysis tool was used to obtain differential mRNAs and miRNAs and screen the differential genes. The standard setting is adj. *p* value <0.01 and |log2 fold change (FC)| > 1. The volcano map and cluster map are used to visually describe the differential expression data.

#### 2.4.2. Target Gene Prediction and miRNA-mRNA Regulatory Network Construction

The target genes of differentially expressed miRNAs were predicted using the TargetScan [11], miRTarBase [12], and StarBase [13] databases. In order to obtain candidate target genes, search for the intersection of target genes predicted by all three databases and GSE108109 differential genes. According to the regulatory relationship between miRNA and mRNA, the miRNA-mRNA regulatory network is constructed. Cytoscape [14] software (version 3.7.2) was used for miRNA-mRNA regulatory network visualization.

#### 2.4.3. Cross-Validation of External Data Sets

The MN-related mRNA expression data set GSE108113 was downloaded from the GEO database. GSE108113 was based on the platform GPL19983 and contained 280 kidney tissue samples, including 5 healthy patients and 87 patients with membranous nephropathy. In order to verify the common genes in the development of MN, we look for the same differential mRNA in the datasets GSE108109 and GSE108113.

#### 2.4.4. miRNA-Regulated Target Gene Function Enrichment and KEGG Pathway Analysis

The WebGestalt [15] online website was used to conduct biological process (BP) enrichment analysis of differential mRNAs in the regulatory network; FunRich [16] software was used to analyze the signal pathway of differential mRNA in the regulatory network.

#### 2.4.5. Candidate Target Gene Protein-Protein Interaction Network Construction

In order to further identify the relationship between candidate target genes, the STRING database [17] is used for protein-protein interaction (PPI), and the Cytoscape software is used for visual analysis of the PPI network. The size of the node is represented by the degree value and is used by CytoHubba [18]. The plug-in MCC [18] algorithm screens out the top 20 core genes and takes the intersection with the target genes in the miRNA regulatory network.

## 3. Results

### 3.1. Differentially Expressed miRNA

Comparing the kidney tissue samples of patients with membranous nephropathy and healthy controls in the GSE51674 data set, 30 differentially expressed miRNAs were obtained, including 22 upregulated (hsa-miR-296-5p, hsa-miR-1249, hsa-miR-1539, hsa-miR-602, hsa-miR-2116∗, hsa-miR-210, hsa-miR-106b, hsa-miR-222, hsa-miR-550, hsa-miR-17, hsa-miR-718, hsa-miR-660, hsa-miR-484, hsa-miR-532-5p, hsa-miR-17∗, hsa-miR-503, hsa-miR-29c, hsa-miR-29a, hsa-miR-27b, hsa-miR-26a, hsa-let-7g, and hsa-miR-24) and 8 downregulated (hsa-miR-29b-1∗, hsa-miR-135a, hsa-miR-126∗, hsa-miR-125a-5p, hsa-miR-30c, hsa-miR-320d, hsa-miR-513a-5p, and hsa-miR-513b); a heat map and volcano map were plotted by using http://www.bioinformatics.com.cn, a free online platform for data analysis and visualization (Figure 1).

### 3.2. Differentially Expressed mRNA

Comparing the kidney tissues of patients with membranous nephropathy and healthy controls in the GSE108109 data set, 1267 differentially expressed mRNAs, including 536 upregulated expressions and 731 downregulated expressions, were obtained. Clustering of the top 50 differential mRNAs with a larger absolute value of the fold change is presented in Figures 2 and 3.

### 3.3. Target Gene Prediction and Regulatory Network Construction

TargetScan, miRTarBase, and StarBase databases were used to predict the downstream targets of differentially expressed miRNAs. Among them, 2957 mRNAs existed in the three databases at the same time (Figure 4(a)), and 2400 miRNA-mRNA relationship pairs existed in the 3 databases at the same time. The intersection of genes and differential genes that exist in the three databases was taken at the same time to obtain 175 candidate target genes (Figure 4(b) and Table 2).

According to the negative regulatory relationship between miRNA and mRNA, 36 miRNA-mRNA relationship pairs consisting of 10 differentially expressed miRNAs and 27 differentially expressed mRNAs were finally screened out. Cytoscape software was used to construct and visualize the miRNA-mRNA regulatory network (Figure 5 and Table 3).

### 3.4. Cross-Validation of External Data Sets

Using the same screening criteria (adj. *p* value <0.01, |log2 FC| > 1), the GSE108113 data set was screened for differential genes; a total of 346 differential genes were screened, of which 121 were upregulated and 225 were downregulated. Compared with the GSE108109 data set, 44 differential genes were found to be upregulated at the same time, and 93 differential genes were downregulated at the same time (Figure 6).

### 3.5. Function Analysis of Network Target Genes

The BP function analysis of differential mRNAs in the regulatory network was carried out through the WebGestalt online website, and a total of 10 entries were enriched, 9 of which were statistically significant, mainly including cellular response to stress, positive regulation of nucleobase-containing compound metabolic process, apoptotic process, positive regulation of RNA metabolic process, response to steroid hormone, negative regulation of DNA biosynthetic process, muscle structure development, regulation of cellular response to stress, and response to organic cyclic compounds (Figure 7). FunRich software was used to analyze the differential mRNA pathways in the miRNA-mRNA regulatory network, which are mTOR, PDGFR-*β*, LKB1, and VEGF/VEGFR signaling pathways.

### 3.6. Construction of Differential Gene PPI Network

The downstream target genes existing in the three databases were intersected with the difference genes in the data set, 175 candidate target genes were obtained, the PPI network was constructed through the STRING database, and the software Cytoscape was used to visually analyze the PPI network graph (Figure 8). The CytoHubba [18] plug-in MCC algorithm was used to screen out the first 20 hub genes (Figure 9(a)), and they were intersected with 27 differential genes in the miRNA-mRNA regulatory network, and finally, 3 hub target genes—NOTCH1, CCND2, and PIK3R1—were obtained (Figure 9(b)). Through the analysis of differentially expressed mRNAs, it is found that NOTCH1, CCND2, and PIK3R1 not only are core target genes but also exist in the miRNA-mRNA regulatory network. Studies have found that upregulation of NOTCH1 can aggravate the degree of renal interstitial fibrosis and the decline of glomerular filtration rate [19]. In addition, RNF152 and TET2 show significantly low expression in the kidney tissue of MN patients. Studies have shown that ring finger protein 152 (RNF152) prevents the activation of mTORC1 by targeting the small *G* protein Rheb, thereby inhibiting the activity of the mTOR signaling pathway [20]. RNF152 can inhibit the activity of mTOR signaling pathway, thereby exerting renal protection. Previous studies have found that abnormal DNA methylation affects gene expression and disease development. Many studies have shown that the pathogenesis of nephrotic syndrome may be related to epigenetic changes [21, 22]. Studies have shown that [23] TET2 regulates DNA methylation and may participate in the occurrence and development of MN by regulating DNA methylation.

## 4. Discussion

With the development of gene sequencing technology and bioinformatics, the types of noncoding RNAs have been continuously improved, and their biological functions have also received increasing attention, which has become a current research hotspot in life sciences. The research on miRNAs has been gradually improved. miRNAs are widely expressed in various tissues and organs of the human body. One miRNA can regulate multiple target genes, and each target gene can be regulated by multiple miRNAs, thus forming a complex miRNA regulatory network. miRNA exists stably in blood, urine, and tissues, and blood and urine miRNAs can be detected without invasive procedures. And the expression in different kidney diseases is relatively specific, so miRNAs may develop into a new marker of MN in the future, which will help diagnose the disease early and evaluate the efficacy.

Although the pathogenesis of IMN is not yet clear, most scholars believe that IMN is an antibody-mediated autoimmune disease. The target antigen located in podocytes is recognized by autoantibodies and combined to form immune complexes deposited on basement membrane podocytes. Under the circumstances, activation of the complement system causes damage and shedding of podocytes, resulting in increased permeability of the basement membrane and a large amount of proteinuria. Studies have shown that a large number of miRNAs have been confirmed to be closely related to the occurrence, mechanism, and prognosis of MN. For example, miRNA-217 [24] promotes podocyte apoptosis by targeting tumor necrosis factor superfamily member 11 and then participates in the occurrence of MN; miRNA-328-5p [25] may participate in MN through inflammation and apoptosis-related pathways such as MAPK-related signaling pathways and p53 signaling pathways; miRNA-186 [10] via Toll-like receptor 4 (TLR4), P2X7, and cysteine caspase-3 participates in the apoptosis of podocytes, leading to increased permeability of the basement membrane, which in turn leads to membranous nephropathy; and miRNA-193a [9] may affect the occurrence of MN by influencing other related factors. Most of the above are focused on the upstream and downstream interactions between a single or several miRNAs/genes/pathways, but the occurrence and development of diseases are the result of a multitarget, multipathway, and multistep synergistic effect. If you only study the relationship between a certain miRNA and gene, it will limit the study of the mechanism of MN to a certain extent.

In this experiment, 22 upregulated miRNAs and 8 downregulated miRNAs were excavated. TargetScan, miRTarBase, and StarBase databases were used to predict downstream targets of differentially expressed miRNAs. It is predicted that 2957 mRNAs exist in the three databases at the same time, and 2400 miRNA-mRNA relationship pairs exist in the 3 databases at the same time. Genes and differential genes that exist in the three databases were intersected at the same time to obtain 175 candidate target genes. According to the negative regulation relationship of miRNA and mRNA, 36 miRNA-mRNA relationship pairs comprising 10 differentially expressed miRNAs and 27 differentially expressed mRNAs are finally screened out. These differential miRNAs and mRNAs may be key nodes in the pathophysiology of MN, and the first 20 core genes are screened out through the CytoHubba plug-in MCC algorithm, and they are intersected with 27 differential genes in the regulatory network to obtain the 3 genes NOTCH1, CCND2, and PIK3R1. Among them, NOTCH1 is significantly highly expressed in the kidney tissue of MN patients. Studies have shown that the degree of glomerular sclerosis and the urine protein level are positively correlated with the upregulation of NOTCH1 expression in renal podocytes, and the upregulation of NOTCH1 in patients with chronic renal failure can aggravate the degree of interstitial fibrosis and the decline of glomerular filtration rate [19].

Through FunRich analysis, it is found that the differentially expressed mRNAs in these regulatory networks are mainly related to mTOR, PDGFR-*β*, LKB1, and VEGF/VEGFR signaling pathways, among which the mammalian target of rapamycin (mTOR) is a highly conserved serine/threonine protein kinase, which is widely present in yeast to animal cells and belongs to the phosphatidylinositol-3-kinase-related kinase (PIKK) protein family [26]. Its stability affects the expression of cytokines in T cells; it participates in immunosuppression, affects transcription and protein synthesis, and regulates cell growth, apoptosis, and autophagy. Studies have shown that autophagy levels in MN patients are abnormal. Animal experiments have found that podocyte autophagy in rats with membranous nephropathy is expressed at a high level, and there is a certain correlation between podocyte damage and shedding and autophagy. A number of studies have confirmed that autophagy is involved in the occurrence and development of MN [27, 28]. The mTOR signaling pathway may participate in the occurrence and development of MN by regulating the autophagy level of cells. The main function of platelet-derived growth factor (PDGF) is to regulate cell proliferation, migration, inflammation, and tissue permeability and participate in extracellular matrix deposition. Chen et al. [29] found that blocking the PDGFR-*β* signaling pathway in a rat model of chronic renal failure can inhibit the progression of renal fibrosis, and some patients with membranous nephropathy will also develop chronic renal failure. Blocking the PDGFR-*β* signaling pathway may be beneficial to the long-term renal prognosis of MN patients. It provides a new treatment strategy for stabilizing the renal function of patients with MN. MN patients are mostly accompanied by dyslipidemia, and lipid metabolism disorders will promote the occurrence and development of the disease. Studies have found that [30] the AMPK-CaMKK*β* (LKB1) signal transduction pathway plays a very important role in lipid metabolism. The LKB1 signaling pathway may affect MN by participating in lipid metabolism. At the same time, MN will eventually lead to renal fibrosis as the disease progresses. Studies have found that vascular endothelial growth factor (VEGF) is an important factor in maintaining the stability of the glomerular filtration barrier structure and the homeostasis of the kidney [31]. Experiments have shown that blocking the VEGF/VEGFR pathway can prevent the transformation of pericytes to myofibroblasts and then delay renal fibrosis [32].

Although the experiment constructed a potential miRNA-mRNA regulatory network based on bioinformatics, there are certain limitations. First of all, the number of kidney tissue cases in the healthy group is relatively small, which may affect the results of the experiment. The main sequencing method is chip sequencing. There is no high-throughput data set. In addition, there is a lack of data sets of the same population and the same platform. Second, the experimental results only involve membranous nephropathy kidney tissue specimens, not urine, blood, and other samples. Finally, the experiment only analyzed gene expression microarrays of membranous nephropathy and did not analyze RNA sequencing data, which lacked the ability to identify new features. In the future, more studies such as the dual luciferase report experiment will be designed to verify the in vivo and in vitro biological functions of the miRNA-mRNA regulatory network model.

In summary, based on the GEO chip data set, with the help of bioinformatics methods, 36 experimental miRNA-mRNA regulatory relationship pairs related to MN were explored and the regulatory network was constructed to clarify the complex network of multiple targets and multiple pathways of MN regulation. The network core targets can improve the clinical performance of MN through mTOR, PDGFR-*β*, LKB1, and VEGF/VEGFR signaling pathways and provide targets and reference directions for further in-depth study of their mechanism of action and treatment of MN.

## Figures and Tables

**Figure 1:** Differentially expressed miRNA kidney samples in patients with MN and healthy patients. (a) Volcano map of differentially expressed miRNAs. Red dots represent upregulation, blue dots represent downregulation, and gray dots represent no differential expression. (b) Heat map of differentially expressed miRNA. Red represents upregulation, and green represents downregulation.

**Figure 2:** Heat map of the top 50 differentially expressed mRNAs with a larger absolute value of the fold change. Red represents upregulation, and green represents downregulation.

**Figure 3:** Volcano map of mRNAs differently expressed in MN. Red dots represent upregulation, blue dots represent downregulation, and gray dots represent no differential expression.

**Figure 4:** Screening of target genes. (a) Venn diagram of TargetScan, miRTarBase, and StarBase databases predicting miRNAs corresponding to downstream target genes. (b) Venn diagram of differentially expressed mRNA and miRNA downstream target genes.

**Figure 5:** MN-related miRNA-mRNA regulatory networks. Red means the expression is upregulated, and blue means the expression is downregulated. miRNA and mRNA are represented by V-shape and circle, respectively.

**Figure 6:** External data set cross-validation Venn diagram.

**Figure 7:** BP enrichment entries of 27 target genes in the miRNA-mRNA regulatory network.

**Figure 8:** PPI network of candidate target genes: red dots represent upregulation, blue dots represent downregulation, and the size of the graph is determined by the degree value.

**Figure 9:** Hub genes and hub target genes. (a) The first 20 hub genes. (b) The first 20 hub genes and they were intersected with 27 differential genes in the miRNA-mRNA regulatory network.

**Table 1:** Databases or software used in this study.

Database/software	URL
GEO database	https://www.ncbi.nlm.nih.gov/geo/
STRING database	https://string-db.org/
TargetScan database	http://www.targetscan.org/vert_72
miRTarBase database	https://mirtarbase.cuhk.edu.cn/
StarBase database	https://starbase.sysu.edu.cn/
WebGestalt database	http://www.webgestalt.org/
FunRich database	http://www.funrich.org/
STRING database	https://string-db.org/
Cytoscape software (3.7.2)	https://cytoscape.org/

**Table 2:** The intersection of mRNAs predicted by differentially expressed miRNAs and differentially expressed mRNAs in MN.

mRNA	LogFC
FSCN1	2.588635
SEMA7A	2.421008
ADM	2.409355
BMP2	2.383218
TNFRSF21	1.945833
NCAM1	1.925172
UCP2	1.909103
TGFB1	1.905343
EGR3	1.847593
BAMBI	1.808341
CCND1	1.743998
CCDC85C	1.655328
ITGA5	1.620048
COL1A2	1.615838
PLD3	1.599157
HBEGF	1.597727
EHD2	1.593748
TRPC6	1.567959
GATA3	1.567876
TP53	1.541281
SKI	1.532832
ST3GAL2	1.511352
PLEKHO1	1.502347
HK2	1.4997
NOTCH1	1.462259
TMEM154	1.430919
PDE4A	1.430186
LYN	1.424265
TMEM184B	1.422096
PLXNC1	1.41303
KPNA2	1.40473
PREX1	1.401679
FAM129B	1.387175
EIF5A2	1.383387
PXDN	1.376657
DAG1	1.371781
FBRS	1.361762
MTSS1L	1.350619
KCTD12	1.34922
RNF44	1.343982
CENPP	1.338335
PRR11	1.335654
VEGFC	1.33485
PCDH17	1.333166
CD248	1.325592
LRP10	1.323391
CCND2	1.320625
ZNF703	1.31591
PLXND1	1.313283
RUSC2	1.312396
COL4A2	1.309219
COL4A1	1.307964
IER3	1.294667
SLIT3	1.29412
GNG2	1.290121
CBX6	1.275551
FKBP14	1.267006
ADAM12	1.255887
EMP1	1.248797
PPM1F	1.247126
ADAMTS1	1.243952
ZCCHC24	1.242563
SEMA4C	1.234261
FN1	1.229458
MARK2	1.218718
SLC35E2	1.213068
ORAI1	1.209795
BTN2A2	1.202712
TMED9	1.201828
KIAA0930	1.200233
PIK3C2B	1.199587
PRR12	1.189574
FICD	1.188868
VASH1	1.18757
CDH5	1.179563
ANK1	1.175622
CDKN1C	1.171323
MAFB	1.160213
NETO2	1.158592
PACS1	1.155518
SLC7A1	1.12978
MAP1B	1.123029
FMNL3	1.120955
NCOR2	1.118047
FOXK1	1.113134
VPS37B	1.109738
SLC35C1	1.104002
CDC42SE1	1.10201
mRNA	logFC
IQSEC1	1.100248
C15orf39	1.099142
STK10	1.098527
MLXIP	1.097227
PDGFRB	1.094398
BCL7B	1.092912
RRM2	1.083712
TNFAIP1	1.082132
RAB23	1.077515
TWIST1	1.077234
KIAA1211	1.075862
TNKS1BP1	1.075735
TRAM2	1.075199
ELK3	1.073763
BAG2	1.073373
BAK1	1.066222
ASB6	1.062721
HID1	1.062155
NFIX	1.04586
PDGFB	1.045391
SYNM	1.043951
KMT2D	1.042489
DTX3L	1.033091
PGM2L1	1.029231
CDK6	1.025282
DDN	1.022429
HYOU1	1.022252
GLTP	1.022145
QSOX2	1.018591
ZNF598	1.017456
LRRC59	1.017138
TNRC18	1.014733
ANKRD52	1.011072
RAB1B	1.002591
EFHD2	1.001892
DUSP1	-1.00608
WNK3	−1.00956
IRF2BP2	−1.00999
SLC38A9	−1.02822
ZFP36	−1.03017
PIK3R1	−1.0368
INTU	−1.04403
HNRNPC	−1.05119
TFRC	−1.07492
LRIG3	−1.08372
MYSM1	−1.08847
PAXBP1	−1.09315
RORA	−1.09921
RND3	−1.10045
IQCB1	−1.1254
SCML1	−1.13556
HNRNPA1	−1.16882
CPM	−1.19419
ACADSB	−1.20615
NEDD9	−1.20698
DDIT4	−1.23395
DDX5	−1.30958
CEBPD	−1.3324
ETNK2	−1.33701
ANK3	−1.34546
RDH10	−1.35602
WSB1	−1.35652
HLF	−1.3639
PFKFB2	−1.36934
ANO3	−1.37338
LUC7L2	−1.40151
OGT	−1.41004
SLC16A9	−1.45495
FKBP5	−1.47532
A1CF	−1.48213
RIMKLB	−1.51655
LUC7L3	−1.52778
GATM	−1.53727
NABP1	−1.5713
ALDH6A1	−1.58547
TET2	−1.59016
RNF152	−1.6183
CHORDC1	−1.67273
SLC4A4	−1.67506
AGMAT	−1.68711
PRLR	−1.84312
IP6K3	−1.90237
EYA4	−1.91033
PDE7A	−1.93011
ANKS4B	−2.13921
GOLGA8A	−2.18853
GOLGA8B	−2.44931

**Table 3:** miRNA-mRNA regulatory pairs associated with MN.

miRNA	Gene symbol	miRNA logFC	mRNA logFC
hsa-let-7g	GATM	1.2	−1.53726793
hsa-let-7g	SLC16A9	1.2	−1.45495451
hsa-let-7g	LRIG3	1.2	−1.08372218
hsa-let-7g	DUSP1	1.2	−1.00608428
hsa-miR-106b	NABP1	3.95	−1.57129602
hsa-miR-106b	SLC16A9	3.95	−1.45495451
hsa-miR-106b	DDX5	3.95	−1.30958254
hsa-miR-106b	RORA	3.95	−1.09920587
hsa-miR-106b	WNK3	3.95	−1.00956193
hsa-miR-125a5p	BAK1	−3.03	1.06622167
hsa-miR-125a-5p	HK2	−3.03	1.49970035
hsa-miR-125a-5p	FAM129B	−3.03	1.38717468
hsa-miR-125a-5p	SEMA4C	−3.03	1.2342607
hsa-miR-17	NABP1	3.5	−1.57129602
hsa-miR-17	SLC16A9	3.5	−1.45495451
hsa-miR-17	DDX5	3.5	−1.30958254
hsa-miR-17	RND3	3.5	−1.10045332
hsa-miR-17	RORA	3.5	−1.09920587
hsa-miR-17	WNK3	3.5	−1.00956193
hsa-miR-24	HNRNPA1	1.12	−1.16881604
hsa-miR-24	SCML1	1.12	−1.13556225
hsa-miR-26a	CHORDC1	1.4	−1.67272568
hsa-miR-26a	TET2	1.4	−1.59015664
hsa-miR-26a	NABP1	1.4	−1.57129602
hsa-miR-27b	EYA4	1.44	−1.91033091
hsa-miR-27b	RNF152	1.44	−1.61830472
hsa-miR-29a	TET2	1.62	−1.59015664
hsa-miR-29a	PIK3R1	1.62	−1.03679898
hsa-miR-29a	ZFP36	1.62	−1.03016982
hsa-miR-29c	TET2	1.77	−1.59015664
hsa-miR-30c	SKI	−3.05	1.5328315
hsa-miR-30c	NOTCH1	−3.05	1.46225942
hsa-miR-30c	CCND2	−3.05	1.32062533
hsa-miR-30c	FOXK1	−3.05	1.1131342
hsa-miR-30c	MLXIP	−3.05	1.09722718
hsa-miR-30c	KMT2D	−3.05	1.04248918

## Data Availability

The simulation experiment data used to support the findings of this study are available from the corresponding author upon request.
